The article "DRG-Oriented Mathematical Calculation Model and Method of Integrated Medical Service Cost" was published in 2020. Journal: Comput Math Methods Med.

# DRG-Oriented Mathematical Calculation Model and Method of Integrated Medical Service Cost

**DOI:** 10.1155/2020/3189676

**Published:** 2020-11-01

**Authors:** Xiaowei Sun, Yi Zhu

**Affiliations:** Jinling Hospital Department of Pharmacy, Nanjing University, School of Medical, Nanjing, 210002 Jiangsu, China

## Abstract

In the context of the new round of medical and health reform, in order to alleviate the problem of “difficult to see a doctor and expensive to see a doctor,” the state focuses on reducing the cost of medical services, so it puts forward the calculation and method research of medical costs. The purpose of this study is to calculate and predict the cost of medical services in a DRG-oriented integrated environment. In this study, activity-based costing and weighted moving average methods are used. First, basic data of medical services are collected, then all medical activities are confirmed and all service costs are collected, then a cost database is established, and a calculation model of medical costs is designed. Finally, calculation suggestions and optimization methods are put forward by analyzing the calculated data. The experimental results show that the actual demand of drugs predicted by the general moving average method is relatively insufficient, with the maximum error of 41%, the minimum of 5%, and the average error of 19.8%; the maximum error of drug demand predicted by the weighted moving average method is 24%, the minimum is 2%, and the average is 15.4%. It can be concluded that the prediction effect of the weighted moving average method is better than that of the ordinary moving average method, which plays a good and effective role in the prediction of medical cost. The activity-based costing method is more detailed and organized for the cost calculation and classification of medical services. It provides a certain value for the effective management and control of medical service cost.

## 1. Introduction

In order to restrain the sharp increase of medical expenses, the method of DRG payment has been adopted internationally. DRG will change the payment based on service items to the payment based on disease types. According to the international disease classification, inpatients are divided into several groups according to diagnosis, etc., to develop the corresponding payment benchmark. What is lower than the price of DRG is the “free profit” obtained by the hospital, and vice versa is the loss borne by the hospital. Therefore, how to effectively manage and control DRG-oriented medical service costs has always been the focus of scholars at home and abroad.

From the existing research, generally speaking, cost prediction and optimal control of medical expenses are limited to individual discussion. The management of medical expenses cannot be dealt with from the overall point of view. At the same time, the existing method and theory of DRG direction of medical service cost management support are insufficient. From a comprehensive perspective, this paper studies the DRG-oriented cost management strategy of medical services, the construction of DRG-oriented general cost management system of medical services, the estimation and optimization control of disease cost, the determination and control of hidden cost, and the total cost of ownership of medical products, further improving the DRG-oriented medical service cost management development of medical service cost management methods and technical system control and medical safety cost management strategy.

About the calculation method of medical service cost, based on the mathematical theory, Szekely proposes a new method to use Benford's law. They carefully check the data at the personal level to determine the specific cost for in-depth analysis. His method is to expand the mathematical theory and prove that large-scale data conforms to Benford's law. Then, they used the actual large-scale medical data of the national patient sample (NPS) of Korea health insurance assessment (HIRA) to test its applicability. For Benford's law, they considered the mean absolute deviation (MAD) formula to test large-scale data; this method cannot predict the budget cost effectively [1]. Hoyle believes that classification systems such as DRG and ICD are the basis of modern medical service planning, capital, operation management, and governance. Existing classification systems, such as ICD, DRGs, and ICF, have evolved for different reasons and reflect unique perspectives on health, disease, care, and “patient therapy.” They proposed a practical method to add patient-centered “dimensions” to the existing classification. For example, they considered the meaning of comprehensive nursing classification from the perspective of ICD/DRG. By adding a dimension to closely link the continuous and stable patient attributes with service integration, they show that it is possible to develop stable and meaningful patient-centered categories across time and space, so as to support patient-centered integration by forging these connections, and the broader nursing integration projects can focus on maximizing and improving the patient's interests rather than being distracted by institutional boundaries. The implementation of this method needs an ideal external environment and various cooperation, and its enforceability is poor [2]. Hardin et al. are mainly engaged in BPCI and cooperate with a group of medical diagnosis-related groups (DRGs). They describe the experience of creating a response system for different personnel and diagnosis in medical DRGs and specifically determine the organizational factors to achieve the successful implementation of bundling. Their experience shows that the interprofessional collaboration program is successful, although it is still in its early stages, and the information observed from their project strategies may provide potential insights for organizations considering participating in BPCI programs. This method is vague and inaccurate in the calculation of medical cost [3].

This study first gives an example of some problems in the current cost management of medical service projects. At the same time, the key technology of DRG-oriented integrated medical service cost management and the composition and classification of medical cost are described. This study also introduces the principle of activity-based costing and the principle of single disease cost prediction based on a support vector machine. Through this principle and weighted moving average method to collect and process data, through the model and calculation method to effectively analyze and predict the medical service cost, the existing scheme is further optimized, so as to better promote the development of DRG-oriented medical service cost management.

## 2. Medical Service Cost and Mathematical Calculation Method

### 2.1. Main Problems in Cost Management of Current Medical Service Projects

At present, the cost management system of many hospitals is relatively chaotic, by which the refining cost management needs of medical service projects are difficult to meet [4].

#### 2.1.1. The Management Did Not Pay Attention to the Cost Management of the Medical Service Project

The cost management of a medical service project is a comprehensive, complex, and human-oriented project. Only when the administrator invests more energy can the unified work instruction be established and play the role of cost management. At present, the hospital management focuses on the calculation of income and cost, but due to the neglect of the supervision of events, the lack of understanding of the control function of management accounting, and the lack of leadership in the cost management of medical service projects, the implementation of detailed cost management is not easy [5, 6].

#### 2.1.2. Weak Cost Management Foundation of Medical Service Project

First, there are insufficient cross-border cost management talents to meet the needs of industry and financial integration. Although the financial director of the hospital has accounting knowledge, he only pays attention to the basic cost calculation and accounting function. Due to the lack of management and evaluation awareness and function of management accounting, the meticulous management of hospital expenses is limited. Secondly, the support of the cost management information system is insufficient. Traditional manual methods cannot meet the needs of cost management; information technology plays an important role in the whole medical system. However, the current hospital information system is not perfect, there is no connection between the systems, and data dispersion, collection, and induction are not easy, which directly affects the accounting and control of medical service cost [7].

#### 2.1.3. The Cost Calculation of Current Medical Service Projects Is More Limited

At present, the cost calculation method of the hospital has fallen behind, most of which are based on departments, which cannot reflect the total cost of the hospital as a whole, and has no contribution to the implementation of refined cost management. At the same time, the cost calculation of the department has fallen into a misunderstanding. First of all, as the benchmark of department bonus using cost calculation, the competition between departments becomes fierce. Secondly, no matter the renewal of machines, investment in scientific research, and other expenses, they will over pursue to reduce costs. Misunderstanding of cost calculation affects the long-term development of hospitals [8].

#### 2.1.4. Imperfect Cost Management and Guarantee Mechanism of Medical Consumables

The cost management of medical consumables is one of the important links in the cost management of medical service projects. According to the survey, the cost of medical consumables in hospitals is increasing year by year, and the proportion of the total cost of medical services is also increasing. According to the price management department, the medical consumables with a unit price lower than 1000 yuan in public hospitals can be increased by 10%. For medical consumables over 1000 yuan, the price increase rate is 8%, and the maximum price increase is 800 yuan. If improper management results in the loss or damage of consumables, the cost of the hospital will rise. Generally speaking, the actual use of consumables in the hospital has been confirmed clinically in the whole process. In fact, the intermediate monitoring link of functional departments does not work, which will lead to not only medical corruption but also waste, directly affecting the decision-making budget of the hospital. Therefore, for the detailed management of medical expenses, it is particularly important to strengthen the construction of a cost management guarantee system of consumables [9, 10].

### 2.2. Key Technologies of DRG-Oriented Integrated Medical Service Cost Management

#### 2.2.1. Disease Cost Prediction Method

Disease cost prediction is the basis of reducing disease cost. The influencing factors of disease cost are distributed in all stages of the process from hospitalization to discharge. The complexity of the disease treatment process will bring many factors and difficult data to cost. At the same time, the importance of factors is very different. Each factor interacts and influences each other. The selection of factors affecting traditional cost is mainly based on experts, lacking theoretical guidance. The detailed estimation method used in traditional cost forecasting needs a lot of time and cost. The parameter prediction method is due to the generalization ability and insufficient adaptability of the model, and the accuracy of cost prediction is not good enough, which almost has no effect on reducing the cost of diseases. At present, a high level of cost prediction method is needed to predict the cost of diseases. The purpose of disease cost prediction is not only to clarify the process of disease cost but also to clarify the inherent law through the analysis of prediction cost and get improved feedback [11, 12].

#### 2.2.2. Disease Cost Control Method

Disease cost management is an important part of DRG-oriented comprehensive medical service cost management. The rationality and scientificity of management methods not only directly affect the effect of hospital cost management but also determine the stability of a hospital operation system. The cost management of disease includes the whole process of disease design, implementation, and improvement, so the cost management of disease must also be implemented through the whole life cycle of disease.

#### 2.2.3. Disease Cost Prediction and Control

The hospital's cost management system is a multioutput service system. The environment of medical service activities is complex, and the cost is affected by various factors. Therefore, there are various reasons for different costs. It is difficult to get satisfactory results with simple statistical tools. The existing disease cost management method usually uses the accounting period as the analysis period. Through the analysis of financial accounting indicators, the medical service process is monitored and controlled. This is usually afterwards management, which has a great impact on the timeliness of cost management. By introducing the idea of predictive control and combining the management chart with artificial intelligence technology, the timeliness of disease cost management can be greatly improved [13].

#### 2.2.4. Cost Difference Identification of Diseases

If we successfully predict and calculate the cost of different kinds of diseases, we need to enable the diagnostic function of different costs to distinguish different types of costs. From the point of view of diagnosis pattern recognition of disease cost difference, according to the principle of management chart, different patterns of disease cost can be divided into six categories: normal, rising trend, falling trend, rising stage, falling stage, and cycle mode. Because the determination of the cost difference of disease is combined with various experiences and knowledge of hospital information systems, it is necessary to make full use of real-time information and knowledge, determine the classification of the cost difference of disease, find out the cause of cost as soon as possible, and take timely countermeasures. The action is adjusting the medical service process to a controlled state [14, 15].

#### 2.2.5. Cost-Oriented Optimization Strategy of Medical Service Operation

The diagnosis system of disease cost difference is only to predict and recognize the disease cost difference, and the specific scheme should be decided by the relevant medical personnel. The allocation of various resources in hospitals directly determines the cost level of diseases. Optimizing the allocation of resources plays an important role in reducing the cost of diseases. In order to cope with the surgical pressure caused by the disease payment system, the introduction of queuing theory of surgical research, mathematical planning and other theories, optimization of hospital facilities, and personnel allocation can greatly reduce the cost of disease [16].

### 2.3. Composition and Classification of Medical Cost

#### 2.3.1. Composition of Hospital Cost

Hospital cost refers to the expenses of various medical services borne by the active TCM hospital. Whether the hospital adopts the former cost usage or the activity-based cost method, the total expenses of the hospital are divided into drug expenses and medical expenses. Medical expenses and material expenses are medical product and material expenses; intangible asset depreciation and fixed asset depreciation required for undertaking in the hospital are fixed asset depreciation and depreciation; wages and welfare expenses used in the hospital of traditional Chinese medicine for intangible assets and medical activities are 5 insurances and 1 fund for basic wages, subsidies, and bonuses, as well as other expenses borne by employees of all departments of the hospital; and management expenses are the daily business and hospital management expenses of the logistics department and management department of the hospital, including business expenses, transportation expenses, travel expenses, and business expenses. In terms of the total cost of the hospital, the proportion of drug and material costs is about 55%, the proportion of wages and welfare costs is about 25%, and the proportion of other costs is about 20%. Shown in Figure 1 is the composition framework of medical service cost [16, 17].

#### 2.3.2. Classification of Hospital Cost

According to different research purposes, hospital cost can be divided into disease cost, project cost, department cost, and hospital total cost. Disease cost refers to the treatment cost of a specific disease, and project cost refers to the expenses incurred in the medical service project. Department cost refers to the daily medical service process in the department to ensure normal operation. The total cost of the hospital refers to the total expenses borne by all departments in the daily operation [18, 19].

Cost can be divided into variable cost and fixed cost according to different forms. Variable cost refers to the total cost of the hospital's business cost and daily business process. The more business, the higher the total cost. The fixed cost has nothing to do with the total cost of the hospital's daily business process. The cost will not change with the increase in transaction volume. A credit card can be divided into indirect cost and direct cost. Indirect cost refers to the cost that cannot be directly included in the cost object. This cost is related to multiple cost objects and needs to be allocated according to the allocation basis, including interest payment, bad debt provision, and lease fee. Direct expenses refer to the expenses that can be directly included in the cost object, such as salary, medicine expenses, and welfare expenses of employees [20].

### 2.4. Principle of Activity-Based Costing

The method of activity-based costing is different from the former costing method. The traditional cost accounting method is limited by the single distribution standard of cost distribution. The allocation method of activity-based cost uses various allocation benchmarks and main principles such as mechanical time and labor force. Consumption resource is operation, product consumption operation, and operation is the intermediate variable between resource and product. In the hospital industry, specifically, patients are registered in the hospital or online, diagnosed, and examined in the outpatient process. These processes are the occurrence of operations, which consume specific resources, and the allocation of product cost based on resource motivation is consumed. The cost calculated by this method becomes more accurate and accurate, and the decision reference value of the manager points up. The activity cost method is widely used in finance, communication, medical, and other fields, and now, it is the main choice of cost management methods for enterprises [21, 22].

### 2.5. Principle of Single Disease Cost Prediction Based on Support Vector Machine

#### 2.5.1. SVM Algorithm

A support vector machine (SVM) is a machine learning method based on statistical learning theory. According to the limited sample data information, the structural risk is controlled to the minimum, and the nonseparable data set is mapped to the high-dimensional feature space. In this way, samples can be distinguished correctly in high-dimensional space, so as to solve the problem of low-dimensional space [23]. The cost estimation of a single disease is related to many factors. It is assumed that *x*_*i*_ ∈ *E* is the factor influencing the cost estimation and *y*_*i*_ is the cost estimation. The steps of single disease cost regression prediction by SVM are as follows.

Set the training sample set of size *L*:

(1) $$\begin{array}{c} \left\{\left(x_{i},y_{i}\right)\left|i=1,2,3,\cdots ,l,x_{i}\in E,y_{i}\right.\in R\right\}. \end{array}$$

Hyperplane in high-dimensional space can be expressed as

(2) $$\begin{array}{c} \omega x+b=0. \end{array}$$

The idea of SVM for inferring regression function is to map the data in input space to high-dimensional feature space through nonlinear mapping *x* and carry out linear regression in high-order element space [24].

SVM uses the following estimation functions:

(3) $$\begin{array}{c} f\left(x\right)=\omega x+b. \end{array}$$

SVM uses the SRM (structural risk minimization) criterion and uses the loss function of *ε* function to measure the risk, which is defined as

(4) $$\begin{array}{c} L\left(y,f\left(x,\delta \right)\right)=L\left({\left|y,f\left(x,\delta \right)\right|}_{\varepsilon }\right). \end{array}$$

The regression estimation problem is defined as minimizing the risk of nonresponse loss function (*ε* ≥ 0). If SVM is used to predict the cost of a single disease, it can be transformed into the minimum value problem of the next convex plan

(5) $$\begin{array}{c} \min\omega \left(a_{i},a_{i}^{*}\right)=0.5{\left(a_{i}-a_{i}^{*}\right)}^{T}K\left(x_{i},x\right)\left(a_{i}-a_{i}^{*}\right)+\varepsilon \overset{l}{\underset{i=1}{\sum }}\left(a_{i}+a_{i}^{*}\right)+\overset{l}{\underset{i=1}{\sum }}\left(a_{i}+a_{i}^{*}\right)y_{i}. \end{array}$$

Among ∑_*i*=1_^*l*^(*a*_*i*_ − *a*_*i*_^∗^) = 0,

(6) $$\begin{array}{c} 0\leq a_{i},a_{i}^{*}\leq C,i=1,2,3,\cdots ,l. \end{array}$$

*K*(*x*_*i*_, *x*) refers to the problem of finding the vector *ω* in a quadratic programming optimization.

In the case of nonlinear separability, for a specific kernel function, any sample in a specific sample group may be the support vector *ω*. General kernel functions include polynomial kernel function, sprite generating kernel function, and radial basis kernel function.

Through the above work, for the cost of a single disease, the SVM regression prediction function can achieve the following results:

(7) $$\begin{array}{c} f\left(x\right)=\overset{l}{\underset{i=1}{\sum }}\omega^{*}K\left(x_{i},x\right)+b=\overset{l}{\underset{i=1}{\sum }}\left(-a_{i}+a_{i}^{*}\right)*K\left(x_{i},x\right)+b. \end{array}$$

In order to use SVM to solve linear and nonlinear regression problems, it is necessary to determine the insensitive value, penalty factor *C*, and kernel function parameters. Choosing different kernel functions will produce different support vectors. This has a great influence on the accuracy of cost estimation. In order to make the RBF kernel function perform well in prediction accuracy and speed, this chapter uses radial basis kernel function RBF:

(8) $$\begin{array}{c} K\left(x_{i},x\right)=\exp\left(-\frac{{\left\|\left(x-x_{i}\right)\right\|}^{2}}{2\sigma^{2}}\right). \end{array}$$

Cost difference analysis and management chart theory also play an important role in disease cost management. The hospital managers and medical staff explained the difference of DRG cost from medical and economic aspects. The hospital is a prolific organization, and the decision of the clinician indirectly affects the cost of the hospital. The target cost of the disease is

(9) $$\begin{array}{c} C=\underset{i,j}{\sum }n\times p_{i}\times r_{ij}\times c_{j}. \end{array}$$

The difference in disease cost is

(10) $$\begin{array}{c} Y=\underset{i,j}{\sum }\left(n\times p_{i}\times r_{ij}\times c_{j}-n^{\prime }\times p_{i}^{\prime }\times r_{ij}^{\prime }\times c_{j}^{\prime }\right). \end{array}$$

#### 2.5.2. Mathematical Calculation Model and Method of Medical Cost

*Simple moving average method*:

(11) $$\begin{array}{c} F_{t+1}=\frac{\sum_{i=t-n+1}^{r}A_{i}}{n}, \end{array}$$

where *F*_*t*+1_ is the demand forecast of time period *t* + 1, *n* is the number of time periods to calculate the moving average (here *n* = 4), *A*_*i*_ is the actual demand in time period *i*, and *w*_*i*_ is the weight in time period *i* (∑*ω*_*i*_ = 1).

*Weighted moving average method*:

(12) $$\begin{array}{c} F_{t+1}=\overset{t}{\underset{i=t-n+1}{\sum }}\omega_{i}A_{i}. \end{array}$$

## 3. Calculation and Treatment of Medical Service Cost

### 3.1. Data Collection and Sorting

The top three collect and check the income data through the hospital information system and financial software. The hospital's expenses are divided into medical expenses, management expenses, and other expenses. In 2019, the total expenditure is 1773122500 yuan, including 15449825475 yuan for medical services and 223297025 yuan for management.

The medical service fee items include Western medicine, traditional Chinese medicine, Chinese patent medicine, and other medicine fee items. There are charging standards for separately charged materials such as cylinder, embedded consumables, vacuum blood sampling needle, oxygen fee, and blood fee, but there is no need for heating fee, diagnosis and treatment fee, incidental fee, application fee, diagnosis and treatment record fee, and external inspection and other medical fees.

As for the department of research and education, it usually does not provide medical services beyond the cost calculation range of pure research-based research institutions in hospitals. In the pharmaceutical sector, there is a special purchasing platform for pharmaceutical products, whose revenue is controlled by the difference between the purchase price and the sales price. The requested item of the pharmaceutical product is not in the cost calculation object. Departments providing services to hospital staff will provide simple diagnosis and prescription services to hospital staff, but this is not included in the cost calculation. As for the special diagnosis and treatment department, the registration fee of the special diagnosis and treatment clinic is different from the usual diagnosis and treatment fee. The diagnosis and treatment are also very simple, and there is no actual implementation project, but the data is very different when calculating the cost of such diagnosis and treatment department.

### 3.2. Medical Cost Calculation Ideas

1. *Collection of Basic Data*. This is done by visiting the hospital, taking the staff of the hospital as the object to conduct a questionnaire survey, first learning the basic medical services of the hospital, then conducting a detailed interview of the hospital, deepening the understanding of the current cost management status and the existing problems of the hospital, and requiring data. Finally, the relevant cost data of the hospital will be collected by category in 2019.
2. *Confirmation Work*. The work flow chart of hospital B shows each process of the hospital, which is composed of multiple operations and summarizes the same operations.
3. *Aggregate Cost: Analyze the Aggregate Cost and Cost Driver*. In the previous cost methods, the current allocation benchmark is used to allocate the related resource cost through the inventory and payable wages recorded in the entry. Cost drivers are based on the nature of resource costs and the types of operations, different for decision.
4. *Build a Cost Library*. A cost library is a collection of similar costs and cost drivers. A cost base can collect management fees and depreciation fees of fixed assets. The number of cost libraries is different from the previous cost accounting, which is the number of cost drivers. It is the benefit of ABC.
5. *Design Model*. After fully understanding the hospital, the mode of the hospital is mainly determined according to the accounting method of operating cost, including confirming the identification and classification of cost objects, resources, and operations; the relationship between different levels; the responsibility of cost objects, cost-driven products, and resources; and the circulation relationship between operations.
6. *Analysis Data*. Analyze the cost data of the hospital under the accounting of activity-based costing.
7. *Put Forward Suggestions*. Put forward relevant suggestions for the problems found in the process of activity-based costing accounting, such as the problem that the cost budget is only in the form and lack of corresponding reward and punishment measures, and improve the relevant organizational structure and establish reward and punishment measures for cost management.

## 4. Calculation Method and Prediction Analysis of Medical Service Cost

### 4.1. Prediction and Analysis of Medical Drug Cost by Moving Average Method

Most medical institutions may have a big error between the future drug forecast and the actual demand. If the patient does not meet the drug demand, it will cause not only economic loss but also mental and physical injury. If the amount of one-time purchase is too much, it will not only restrict the flow and direction of funds but also lead to the overall rise of various related costs (the largest of all costs including procurement costs). Excess inventory is also easy to lead to the omission of custody and management.

The best way to forecast demand is to compare and analyze, collect and sort out the past consumption data (available and accurate) according to the four main factors (season, trend, cycle, and random) of forecast, follow this rule, and establish economic order quantity (EOQ) which is a single order quantity that can minimize the total order cost, storage cost (including holding cost), and economic loss caused by insufficient inventory. Only with accurate demand forecast can we realize the best combination of demand and supply on all links of the supply chain and reduce and avoid the phenomenon of affecting clinical business due to rebate, waste, or shortage.

From January 2019 to December 2019, the number of sales boxes of regional health service centers located in Dongcheng District of Beijing is as follows. It can be calculated by the simple moving average method. The drug demand forecast is from January 2019. As shown in Table 1, the dynamic average method forecasts the demand for drugs.

Figure 2 shows the comparison between the actual demand and the predicted demand. As can be seen from Figure 2, the predicted demand for the drug was generally high in the first half of the year, while it was generally low in the second half of the year, and the highest demand reached 58 boxes in December, which may be caused by more diseases caused by severe cold weather. It can be seen from the trend and fluctuation of the error curve in the figure that there is still a little shortage in predicting the actual demand of drugs, with the maximum error of 41% and the minimum error of 5%, among which the average error of 19.8%. This result is relatively general for the prediction of drug use, and it can have a certain effect, but the effect is not good. This also makes the hospital have a certain deviation in the medical cost of purchasing drugs.

### 4.2. Prediction and Analysis of Medical Cost by Weighted Moving Average Method

Figure 3 shows the prediction of drug demand by the weighted moving average method.

It can be seen from Figure 3 that after the weighted moving decomposition method for drug demand prediction, the result is relatively good. It can be seen from the curve trend that the fitting degree of actual demand and forecast demand curve is quite high, especially at the beginning of the year with high demand, and in the year with low demand, the forecast effect is good. From the error curve, the highest is 24%, the lowest is 2%, and the average is 15.4%. It can be concluded that the prediction effect of this method is better than that of the ordinary moving average method. It plays a good role in the prediction of medical cost.

When the weighted moving average method is used to predict the result, the value of the tracking signal is 55.2%. Such a big mistake may be due to improper weight selection, so the weight will be reselected for calculation, but the result will be further deteriorated. The reason for this big mistake is that it is not appropriate to select the weight, or after selecting parameters from the horizontal direction, you need to specify the weight separately.

### 4.3. Calculation and Analysis of Medical Cost by Activity-Based Costing

The business cost, indirect cost, health material cost, and other expenses included in the inspection activity cost are related to the number of cases of medical service, so the number of cases of each medical item inspection can be calculated according to the number of cases. As shown in Figure 4, the distribution of health material cost is based on activity-based costing.

As shown in Table 2, the distribution table of health material cost is given.

It can be seen from Figure 4 that in the cost of health materials, other costs account for more than 7000 in total, and the cost of each of the seven projects is different, including the highest cost of obstetrics and the lower cost of thyroid and neck blood vessels. It can be concluded that activity-based costing is particularly clear in the calculation and statistics of medical service cost.

### 4.4. Comparative Analysis of Medical Cost Calculation Methods

Based on the improved SVM data mining method, the DRG disease series cost prediction method, its objective data, prediction accuracy, and speed will become higher. The prediction results can be used as a reference value for the cost of new disease cases. Doctors not only modify the treatment plan to reduce the cost, so that the hospital can correctly grasp the future cost level and change trend, but also formulate the cost optimization control standard to provide a scientific and intuitive basis for the decision of hospital management. The model fully considers the multifactor, nonlinear characteristics of disease cost and the similarity of medical service composition of each case. According to the improved SVM proposed DRG disease series cost prediction model, it can be reused. After obtaining the new instance, we can directly use the influence factor information to predict the cost according to the specific value of the disease instance with the minimum condition attribute set in the model.

As shown in Figure 5, the ROC chart of the medical cost prediction algorithm is shown.

According to Figure 5, our algorithm is superior to the BP algorithm and SVM algorithm in the prediction of medical cost. The results show that this method is effective and excellent and can obtain effective knowledge which is directly used on the basis of knowledge. Therefore, this method has a wide range of application prospects in the DRG direction of disease cost prediction. It can provide an effective auxiliary means for the cost prediction of single disease and DRG disease series and has important theoretical and practical significance.

The prediction curve and actual curve using three methods are shown in the figure. The calculation time of the BP neural network, standard SVM algorithm, and white paper algorithm is 15.97 seconds, 10.32 seconds, and 5.71 seconds, respectively. Compared with the BP neural network and SVM algorithm, our algorithm can greatly improve the accuracy and speed of prediction, so it has a better application prospect in the field of DRG disease series cost prediction.

## 5. Conclusion

In order to give full play to the role of medical expense management in hospital management and solve the problems and defects in the implementation of DRG in China, this chapter combines the idea of comprehensive management to study the structure of DRG-oriented comprehensive medical expense management. This paper puts forward the management characteristics, DRG-oriented integrated medical service cost management mode, and its structure chart and investigates the characteristics and problems of disease cost prediction and control under the integrated medical service cost management mode in detail.

This study discusses the structure and function of DRG-oriented integrated medical service cost management, constructs the theoretical framework of DRG-oriented integrated medical service cost management mode, and constructs the framework of DRG-oriented integrated medical service cost management mode. The model describes the structure and characteristics of the system framework in detail. The basic theory of DRG-oriented comprehensive medical service cost management is complete. Due to the introduction of the DRG-oriented integrated medical service cost management mode for a relatively short time, the basis of previous research is relatively weak, especially the composition of the framework and the principles of the implementation framework, which needs further theoretical research.

In the DRG payment system, medical service cost management has become an important means for hospitals to successfully implement the DRG payment system and improve their economic and social interests. However, the current cost management of medical services is basically limited by cost calculation, and the scope of the management concept is very narrow. This study summarizes and analyzes the impact of DRG on the cost management of medical services and the main cost management issues of DRG in the process of hospital introduction in China. DRG is studied from the perspectives of cost, hidden cost, financing cost, and medical safety cost. The general medical cost management strategy promotes the development of DRG-oriented medical cost management, further improves and perfects the theory of medical cost management, and provides guidance for hospitals to improve the level of medical cost management.

## Figures and Tables

**Figure 1:** Structure of medical service cost.

**Figure 2:** Comparison between actual demand and predicted demand.

**Figure 3:** Prediction of drug demand by the weighted moving average method.

**Figure 4:** Distribution of health material cost based on activity-based costing.

**Figure 5:** ROC chart of the medical cost prediction algorithm.

**Table 1:** Prediction of drug demand by the moving average method.

Month	Actual demand (box)	Forecast demand (box)	Error	Error rate
1	50	46	4	8%
2	36	48	-12	34%
3	45	47	-2	5%
4	34	48	-14	41%
5	29	40	-11	36%
6	18	24	-6	33%
7	31	38	-7	22%
8	45	40	5	11%
9	43	38	5	13%
10	38	34	4	9%
11	46	39	7	14%
12	58	44	14	25%

**Table 2:** Distribution of health material cost.

Project	Number of cases	Cost of health materials	Cost of operation	Other expenses
Digestive system (P1)	946	505.96	1011.92	10703
Urinary system (P2)	1532	398.32	796.64	8426
Gynaecology (P3)	2420	629.2	1258.4	13310
Obstetrics department (P4)	5978	1554.28	3108.56	32879
Breast (P5)	1624	422.24	844.48	8932
Thyroid (P6)	558	145.08	290.16	3069
Neck vessels (P7)	604	157.04	314.08	3322

## Data Availability

No data were used to support this study.
